# Removal of Pb (II) Ions from Aqueous Solutions by *Cladophora rivularis* (Linnaeus) Hoek

This article has been retracted.

**DOI:** 10.1100/2012/793606

**Published:** 2012-05-03

**Authors:** Naser Jafari, Zoreh Senobari

**Affiliations:** Department of Biology, Faculty of Basic Sciences, University of Mazandaran, Babolsar 11252, Iran

## Abstract

Biosorption of Pb(II) using *Cladophora rivularis* was examined as a function of initial pH heavy metal concentration and temperature. The optimum pH value for the biosorption of lead was 4.0. The adsorption equilibriums were well described by Langmuir and Freundlich isotherm models and it was implied by the results that the *C. rivularis* biomass is suitable for the development of efficient biosorbent in order to remove Pb(II) from wastewater and to recover it. The high values of correlation coefficient (*R* ^2^ = 0.984) demonstrate equilibrium data concerning algal biomass, which is well fitted in Freundlich isotherms model equations. The dimensionless parameter *R*_L_ is found in the range of 0.0639 to 0.1925 (0 < *R*_*L*_ < 1), which confirms the favorable biosorption process. Fourier transform infra-red (FTIR) spectroscopy of *C. rivularis* was used to reveal the main function groups of biosorption, which were hydroxyl, amine groups, C–H stretching vibrations of –CH3 and –CH2, and complexation with functional groups. All these results suggest that *C. rivularis* can be used effectively for removal of Pb(II).

## 1. Introduction

Industrial pollutants are full of heavy metals, which are harmful to humans and other forms of life and their toxic outlook has a strict environmental impact. This is the consequence of carrying out severe laws regarding to the maximum permissible (authorized) limits of industrial effluents straight into open landscapes and water bodies. Lead, as a raw industrial material, is used for the purposes of storage battery manufacturing, pigments, printing, photography materials, fuels, and explosive manufacturing [1]. Pb(II) is a strong neurotoxic metal, so the pollution of this material is of high concern. The occurrence of lead in drinking water, however, in low concentrations, may cause diseases such as anemia, hepatitis, and nephrite syndrome [2]. There are much information with reference to the biosorption of lead metal ion on marine algae [3, 4], green seaweed [5], and freshwater green algal species [6], with unreliable removal of efficiencies, maximum adsorption capacities (*q*_max⁡_), and binding constants. *Cladophora rivularis* is a green filamentous algae among the algal biomass used for biosorption, which is an easily accessible resource of biomass for the reason of heavy metal removal from wastewater. Experiments carried out by several researchers established the fact that *Cladophora* sp. is competent and capable of accumulating heavy metals such as chromium and zinc [7–9], but there are still a lot of reachable opportunities to use it through available large quantities of algae for the removal of other heavy metal ions from wastewater and sewage system. Biosorption investigations relevant to the removal of Pb metal ion from waste water by means of *Cladophora* sp. are conducted in the same series of this study. The adsorption isotherms and the obtained results, on comparing its adsorption capability with some other adsorbents, indicated that it is the most suitable and fitting material in developing a biosorbent of high competency for the process of Pb(II) removal. *Cladophora* are large group of marine benthic algae. They offer several advantages for biosorption because of their larger surface area.

The goal of the present study is to examine the efficacy of various kinds of locally available biomass in order to remove Pb(II) from aqueous environments. Many studies have shown that algae have a high metal-binding capacity [10] because of the polysaccharide groups, which exist in the cell walls of the algae and can act as binding sites for metals.

## 2. Material and Methods

### 2.1. Chemicals

All of the chemicals used in this experiment acquired an analytical grade, which was obtained from Merck, Germany. A stock solution of lead was prepared in double-distilled water using lead nitrate and the purified water was primed by means of a Millipore Milli-Q water purification system. Pb(II) solutions of different concentrations were produced through diluting the stock solution and the standard Pb(II) solution (1000 mg/L) with regard to the atomic absorption spectrophotometer was achieved from Merck, Germany. In addition, standard acid and base solutions were used for pH adjustments.

### 2.2. Equipment

 pH measurements were done using a pH meter. An atomic absorption spectrophotometer model Z-7000 at a wavelength of 283.3 nm was used in order to analyze the lead solutions and a LEO 435 VP was utilized for means of scanning electron microscopy. Carbon content was measured by an Elementar CHNS analyzer model Vario EL III. TGA studies were conducted on Perkin Elmer in the temperature range 20–750°C besides. FT-IR spectroscopy was used to detect vibration frequency change in the *C. rivularis *biomass. The spectra were collected by FTIR Perkin Elmer model-1600 spectrometer within the range 400–4000 cm^−1^ using a KBr window. The background obtained from the scan of pure KBr was automatically subtracted from the sample spectra. All spectra were plotted using the same scale on the transmittance axis.

### 2.3. Biosorbent

The fresh algal biomass, which was obtained from Caspian Sea on Babolsar city near the University of Mazandaran, was washed with distilled water before use, in order to remove dent, a filter paper was needed to be used to keep the algal biomass in it for reducing the water content. Then, the biomass was dried under direct sunlight for 4 whole days that was followed by drying in an oven at the temperature of 70°C for a period of 24 hours and then ground on an agate stone pistol mortar. Finally, the biomass was sieved in order to select the particles between the mesh size of 150 and 250 to be used.

### 2.4. The Effect of Solution pH on Heavy Metal Adsorption

The influence of pH on Pb(II) adsorption was studied through using 2 g/L of biosorbent and a series of 1 mmol/L of Pb(II) solutions. The pH of the Pb(II) solutions was adjusted from 2.0 to 8.0 by 0.1 mol/L HNO_3_ or by 0.1 mol/L NaOH and the pH adjustments were maintained during the experiment. The blank samples without any biomass were used as controls. In addition, the mixtures were shaken on a rotary shaker for up to 6 hours in room temperature (25 ± 1°C) and then left constant to reach the needed balance and stability and then were filtered through an acid-cleaned 0.45 *μ*m millipore filter. The absorbent was removed and the filtrates then were analyzed using flame atomic absorption spectrometry.

### 2.5. Adsorption Isotherm

 During biosorption, a rapid equilibrium is established between adsorbed Pb(II) ions on the algal cells (*q*_eq_) and unadsorbed Pb(II) ions in solution (*C*_eq_). This equilibrium can be represented by the Langmuir or Freundlich adsorption isotherms, which are widely used to analyze data for water and wastewater treatment applications. The Freundlich equation model is expressed as

(1) $$\begin{array}{c} q_{\text{eq}}=K_{F}\;{C_{\text{eq}}}^{1/n}. \end{array}$$

In this model, *K*_*F*_ (L g^−1^) and 1/*n* are the constants, which are to be determined from the data. In good absorbents, the 1/*n* constant is between 0.2 and 0.8 and a smaller value of 1/*n* indicates better adsorption and formation of rather strong bond between the adsorbate and absorbent.

Here is the Langmuir equation:

(2) $$\begin{array}{c} q_{\text{eq}}=\frac{q_{\max}b\;C_{\text{eq}}}{1+b\;C_{\text{eq}}}. \end{array}$$

In this relation, *q*_max⁡_ (mg g^−1^) stands for the amount of adsorption corresponding to complete monolayer coverage. In other words, *q*_max⁡_ is the maximum adsorption capacity, and *b* (L mmol^ −1^) is the Langmuir constant.

The essential characteristics of Langmuir isotherm can be explained in terms of dimensionless constant separation factor (*R*_*L*_) which is expressed as

(3) $$\begin{array}{c} R_{L}=\frac{1}{\left(1+bC_{0}\right)}. \end{array}$$

The values of *R*_*L*_ from the different initial concentrations used are between 0 and 1 for a favorable biosorption, while *R*_*L*_ > 1 represents an unfavorable biosorption, and *R*_*L*_ = 1 represents the linear biosorption, while the biosorption operation is irreversible if *R*_*L*_ = 0 [11].

## 3. Results and Discussion

### 3.1. Effect of Solution pH on Heavy Metal Adsorption

pH is a very important parameter that affects any biosorption procedure. It affects the activity of the functional groups present in the biosorbent that are accountable for metal adsorption and affects the competition of metallic ions to be adsorbed to the active sites [12]. The pH optimization study was carried out for the removal of Pb(II), using *C. rivularis* in the pH range of 2.0–8.0. The result is presented in Figure 1. The Pb(II) removal positively correlates with the pH of up to 4.0 and then remains practically constant. Therefore, pH 4.0 was considered as the optimum pH for adsorption by *C. rivularis* and the percentage of adsorption was approximately 97%. Comparable values of optimum pH for sorption of Pb are reported in the literature using cone biomass of *P. sylvestris* [13] and pH 5.0 using maple sawdust [14] and activated sawdust [15]. The reduction of adsorption capacity of *C. rivularis* at lower pH can be credited to the competition faced by Pb(II) ions with H^+^ ions to get adsorbed on the binding sites of the cells, which are accountable for metal adsorption [15]. The results showed strong pH confidence of biosorption. This is reliable with the results obtained for the other adsorbent systems [16, 17]. The cell wall matrix of green algae contains complex heteropolysaccharides that can provide amino, carboxyl, and sulphate groups [18, 19]. At low pH, cell wall ligands are protonated and confine the approach of metal actions because of the repulsive force. As pH increases, more ligands such as amino, phosphate, and carboxyl groups would be exposed and carry negative charges with subsequent desirability of metal ions [20]. Tien [6] also observed that the pH was the most important aspect affecting the biosorption of lead, with the optimal values occurring between 4.0 and 5.0. Therefore, the burly pH dependence of Pb(II) biosorption observed in this study could be qualified to more pronounced electrostatic attraction taking place between the biosorbents and the metal ions at higher pH. 

### 3.2. Effect of Temperature on Adsorption

The relationship between percentage removal and contact time and different algal dose (5, 10 and 15 g/L) and relationship between percentage removal and contact time at different temperatures, that is, 30, 40, 50, and 60°C, respectively, at normal pH and optimum algal dose of 5 g/L is given in Figures 2 and 3. After 30 min, thermal equilibrium was achieved and the percentage of removal of Pb(II) decreased from 81 to 45 percent with increase in temperature from 30–60°C. At optimum temperature (30°C), percentage removal ranges between 83–87 percent for different contact time (30–180 min). An increase in the biosorbed amounts with increasing temperature from 30–40°C deals with an increase in the biosorption capacity of biomass. Further increase in temperature from 40°C may change the surface activity of biomass resulting in a decrease in removal value, indicative of that this process is exothermic in nature. The present results showed no thermal deactivation of biosorption activity under operational temperatures. Consequently, the used organisms could acclimatize to wide range of temperature.

### 3.3. Adsorption Isotherms

 The Freundlich isotherms constants having a high value of *n* give an idea of whether the sorption intensity is favorable over the entire range of concentrations tested or is favorable only at high concentrations [21]. The Freundlich isotherm constants were given in Table 1, the magnitude of Freundlich exponent (*n*) showed that adsorption is good, which is again suggestive of a favorable sorption process [22]. It can be concluded that *C. rivularis *has the probable to be used as an effectual and economic biosorbent material for removal and recovery of Pb(II) from wastewater.

In batch adsorption studies, data show that dried *Cladophora rivularis *has considerable potential for the removal of metal ions from aqueous solution. The Freundlich adsorption isotherm model fitted very well with studied metal concentration ranges at 30°C. It is found that the values of correlation coefficients *R* ^2^ obtained from the Langmuir isotherm are from 0.861 to 0.952 which is lower than that from Freundlich isotherm as given in Table 1. The dimensionless parameter *R*_*L*_ is found in the range of 0.0639 to 0.1925 (0 < *R*_*L*_ < 1), which confirms the favorable biosorption process. Although the Langmuir isotherm is widely used, the obtained result indicates that the equilibrium data is not fitted well with the Langmuir isotherm. The Freundlich isotherm shows the best fit to the experimental data with good correlation coefficients (0.963–0.984) compared with Langmuir biosorption isotherms. This result indicates that the uptake of Pb(II) occurs on a heterogeneous surface by multilayer biosorption. The values of *K*_*F*_ are found to increase with increasing temperature, which suggests the biosorption process is endothermic.

### 3.4. Fourier Transform Infrared (FT-IR) Analysis

 The prominent binding sites can be identified by comparing the pristine biomass with that of the metal adsorbed one. The FT-IR spectrum of the pristine biomass and loaded with Pb(II) was shown in Figure 4. Various researchers have suggested that different chemical functional groups such as carboxyl, hydroxyl, and amide are responsible for biosorption of metal ions [23, 24]. These functional groups are the potential sites for adsorption and the uptake of metal depends on various factors such as abundance of sites, their accessibility, chemical state, and affinity between the adsorption site and metal. The FTIR spectroscopy is an important analytical technique, which detects the vibration characteristics of chemical functional groups that are present on adsorbent surfaces. Some intense characteristic bands were obtained from the functional groups presented in proteins and polysaccharides. FTIR spectra of native *C. rivularis* (Figure 4(a)) show sharp peak at 3620, which represented the peak of stretching vibration of free (non hydrogen-bonded) O–H and broad peaks between the region 3500 and 3200 cm^−1,^ which represented the overlapping peaks of stretching vibration of O–H and N–H groups [24–26]. The region between 3000 and 2800 cm^−1^ exhibited the C–H stretching vibrations of –CH_3_ and –CH_2_ functional group. The acrylamide I (–C=O stretching vibration) and acrylamide II bonds (N–H bending vibration and C–N stretching vibration) were prominent at 1654 cm^−1^ [25–27]. The principle amide I absorption peak at 1654 cm^−1^ is mainly accounted for by the 3-helical structure of proteins, although, amino sugar have also a strong absorbance in that region [27]. The strong absorption peaks between 1,000 and 1,100 cm^−1^ also ascertained the presence of carboxyl groups in the polysaccharide structure [27]. Peaks at 1300–1470 cm^−1^ were the deformation stretching of C–H, –CH_3_ and –CH_2_ functional groups. The strong band within 1100–1000 cm^−1^ is due to C–O group, which is the characteristic peak for polysaccharides [24]. Changes in intensity and shift in position of the peaks could be observed in FTIR spectrum after Pb(II) adsorption on *C. rivularis* biomass (Figure 4(b)). The first change was the disappearance of peaks at 3620 cm^−1^ and enhancement of the intensity at the region 3500–3200 cm^−1^, indicating decrease of free –OH and an increase of the hydrogen bonded hydroxyl group on the biomass. The shifting of peak at 1654 to 1651 cm^−1^ indicates the involvement of N–H of amines and C–O of amides in the adsorption process [24]. The minor shift of the peak from 1032 to 1031 cm^−1^ also suggests the involvement of C–O group in binding Pb(II). It is clear from the FTIR analysis that the possible mechanism of adsorption of Pb(II) on *C. rivularis* biomass may be due to physical adsorption and complexation with functional groups and chemical reactions with surface sites.

## 4. Conclusions

*Cladophora rivularis *as a sort of biosorbent was investigated for the removal of Pb(II) from aqueous solutions. It was observed that the biosorption was highly dependent on pH. The biosorption capacity increased as the initial concentration of Pb(II) in solution and temperature increased. The equilibrium biosorption data were best fitted with the Freundlich isotherm which confirmed the multilayer biosorption mechanism of Pb(II) on a heterogeneous surface. The FTIR spectrum of *C. rivularis *has shown a clear difference in natural and Pb(II) loaded forms. The biosorption of Pb(II) was mainly due to Pb(II) bound on hydroxyl, amine groups, C–H stretching vibrations of –CH_3_ and –CH_2_ and complexation with functional groups. All these results suggest that *C. rivularis *can be used effectively for removal of Pb(II).

## Figures and Tables

**Figure 1:** Effect of pH on sorption of Pb(II) by *C. rivularis*.

**Figure 2:** Effect of contact time on the sorption of Pb(II) by *C. rivularis* at natural pH.

**Figure 3:** Effect of temperature on percent removal of Pb(II) at different contact time by *C. rivularis. *

**Figure 4:** FTIR spectra of *C. rivularis* biomass: (a) native, (b) Pb (II) loaded.

**Table 1:** Isotherm constants for Pb(II) biosorption by *C. rivularis. *

Initial Pb(II) concentration (mg/L)	Freundlich			Langmuir		
	*n*	*K*_*F*_ (L g^−1^)	*R* ^2^	*q*_max⁡_ (mg g^−1^)	*b *(L mmol^−1^)	*R* ^2^
1	2.123	6.121	0.963	12.064	0.224	0.861
5	3.261	11.326	0.965	48.136	0.140	0.952
10	3.146	12.065	0.984	37.036	0.521	0.891
15	2.242	8.915	0.965	22.228	0.162	0.883
